This article has been retracted.

# An empirical analysis of the impact of gender inequality and sex ratios at birth on China’s economic growth

**DOI:** 10.3389/fpsyg.2022.1003467

**Published:** 2022-10-26

**Authors:** Xuehua Wu, Arshad Ali, Taiming Zhang, Jian Chen, Wenxiu Hu

**Affiliations:** ^1^Shenzhen Strong Sports & Health Management Center, Shenzhen, China; ^2^Department of Economics and Finance, Greenwich University, Karachi, Pakistan; ^3^Business School, University of Edinburgh, Edinburgh, United Kingdom; ^4^Faculty of Social & Historical Sciences, University College London, London, United Kingdom; ^5^Center of Population and Development Policy Studies, Fudan University, Shanghai, China; ^6^Postdoctoral Research Workstation, China Everbright Group, Beijing,China

**Keywords:** gender inequality, sex ratio at birth, female labor participation, economic growth, China

## Abstract

The contribution of women to China’s economic growth and development cannot be overemphasized. Women play important social, economic, and productive roles in any economy. China remains one of the countries in the world with severe gender inequality and sex ratio at birth (SRB) imbalance. Severe gender inequality and disenfranchisement of girls with abnormally high sex ratios at birth reflect deep-rooted sexism and adversely affect girls’ development. For China to achieve economic growth, women should not be ignored and marginalized so that they can contribute to the country’s growth, but the sex ratio at birth needs to be lowered because only women can contribute to growth. Thus, this study empirically predicts an asymmetric relationship between gender inequality, sex ratio at birth and economic growth, using NARDL model over the period 1980–2020. The NARDL results show that increases in gender inequality and sex ratio at birth significantly reduce economic growth in both the short and long term, while reductions in gender inequality and sex ratio at birth significantly boost economic growth in both the short and long term. Moreover, the results show the significant contribution of female labor force participation and female education (secondary and higher education) to economic growth. However, infant mortality rate significantly reduced economic growth. Strategically, the study recommends equal opportunities for women in employment, education, health, economics, and politics to reduce gender disparities and thereby promote sustainable economic growth in China. Moreover, policymakers should introduce new population policy to stabilize the sex ratio at birth, thereby promoting China’s long-term economic growth.

## Introduction

Knowing the word “inequality,” there are many opinions and it may be an important factor in causing widespread social ills, such as health inequalities, educational disadvantage, crime, and intergenerational mobility, which can weaken social cohesion. It conveys economic execution in a more complex way than the simple trade-off between inequality and economic growth (Amaro et al., 2021). Societal productivity is constrained, and ultimately the process of economic growth is slowed by persistent inequality, causing the economy to pay the price for current declines in productivity and future declines in national output (Jackson, 2019). Since the early 1980s, a central policy issue has been the increase in income and household income inequality (Cevik and Correa-Caro, 2020; Costantini and Seccareccia, 2020; Therborn, 2020).

Global income inequality has widened as a result of the recent COVID-19 pandemic, especially in emerging economies such as China, both within and between countries, setting back progress by a decade or more. Low-income vulnerable groups, such as women, youth, and informal workers face severe income loss and severe unemployment. Women and informal workers in China have higher levels of inequality in terms of access to health care and education, as well as the scale of income loss and jobs due to COVID-19 (World Bank, 2022). China’s development goals will be missed as Chinese policymakers face a clearly faltering economy, a challenge compounded by China’s persistent inequality (Chung et al., 2021). The number of workers flowing into the less secure informal economy has risen sharply due to changes in the labor market, while employment in China’s formal manufacturing sector is declining. In China, many employees lack the competencies needed to perform high-skilled and high-wage jobs, and this inequality continues in education and health care as the Chinese economy seeks to reach high-income status (CSIS, 2022). The Gini coefficient values calculated by the National Bureau of Statistics (NBS) and the China Family Group Study (CFPS) in the graph below are higher than other countries and continue to rise (see Figure 1).

**Figure 1:** China’s inequality is on the rise, estimated by the Gini coefficient. Source: National Bureau of Statistics of China and National Bureau of statistics.

Gender issues are often excluded from empirical studies of data collection design and planning at the micro and macro levels, although this is acknowledged by both academia and policy. Opportunities for different activities, roles, responsibilities, and constraints are disproportionately analyzed for women compared to men (Ho and Maddrell, 2021). As can be seen from the literature, women are still devalued due to prevailing cultural beliefs in China (Wang and Keane, 2020). Household heads spend more on food, with female heads of households spending more, while analyzing gender inequality (O'Brien et al., 2016; Nwaka et al., 2020). Likewise, women are often perceived as lacking elements of wealth, such as buildings, land, investments, and other valuable possessions. In fact, widows lose extraordinary wealth with the death of their husbands because of the local culture. The majority of the female population is engaged in buying and selling, and there are also retired, unemployed and students, of which 20% are engaged in agriculture and industry, while the majority of men are engaged in industry and agriculture. The inequality of femininity in terms of education, health, income resources, family, and other life-enhancing infrastructure makes them completely perceived as absolutely poor. At a time when growth is already slowing, the widening gender gap in China’s labor market—if it persists—could become an even bigger burden on the economy. China’s rise as a global economic power over the last few decades has put women at a disadvantage and worsened gender inequality in its workforce. China’s rise as a global economic powerhouse over the past few decades has disadvantaged women and exacerbated gender inequality in the workforce. Female labor force participation rates have fallen to low levels by international standards, gender pay gaps and gender discrimination are pervasive in the labor market, and there is evidence of growing prejudiced perceptions of women’s rights at work and workplace leadership (PIIE, 2020). Several studies such as Kvangraven (2021), Leach et al. (2021), Omar and Inaba (2020), and Van et al. (2021) have highlighted inequalities in various dimensions, such as trade, financial systems, societies, economies, and reliance on economic interrelationships between the experiences of developing and developed countries. One of the issues of gender preference in China is son preference. An attitude that can explain a preference for sons, a belief that girls are less valuable than boys, can also be defined as gender bias (Wang et al., 2020). “Women hold up half the sky” is an old Chinese saying, which means that Chinese families prioritize sons over daughters. So, like many of its neighbors, millions of missing women are currently facing China (Tian and Bush, 2020). Patriarchal preference is an ancient trait and is often considered a new phenomenon in Chinese society. Due to the one-child policy of 1979 and widespread infanticide, the sex ratio of boys and girls has become unbalanced (Jiang and Zhang, 2021). In general, the higher the death rate, the higher the proportion of boys born naturally, but in China, girls receive less medical care during childhood and are more likely to be neglected than boys (Wan et al., 2020). The introduction of the one-child policy and sex-selective abortion further reinforced this unequal ratio. Around 1985, with the implementation of the one-child policy, sex selection techniques spread in China. The sex ratio at same-day births rose sharply, allowing researchers to decide whether to continue using these methods based on the sex of the fetus. According to the National Bureau of Statistics of China (2020), China’s male population exceeds the female population by more than 30 million, facing a huge gender imbalance. The data show that in 2019, the sex ratios at birth (males to 100 females) of children aged 10–14 and 15–19 were the most unbalanced in China, at 119.10 and 118.39 respectively, which means that there are about 120 males for every 100 females. Birth rates are also likely to decline, as gender imbalance will lead to a marriage crisis within 20–30 years, especially in remote, rural, and poor areas. The sex ratios for 20–24 and 25–29 years were 114.61 and 106.65, respectively, indicating that at least one in 11 men could not marry a woman of the same age. China remains one of the countries in the world with a severe imbalance in the sex ratio at birth (SRB). The disenfranchisement of girls with such abnormally high levels of SRB reflects deep-rooted sexism that adversely affects girls’ development (UNICEF, 2021).

Gender inequality and high sex ratio at birth in China clearly reflect social neglect of women leading to economic underdevelopment. Therefore, this study aims to explore how reducing gender inequality and stabilizing a high sex ratio at birth (male to 100 females) can boost China’s economic growth. Most studies have examined the separate linear effects of these two variables (gender inequality and high sex ratio at birth) on economic growth; however, we were unable to find nonlinear effects of both variables on economic growth at the same time. The non-linear effects of gender inequality and sex ratio at birth on economic growth suggest that an increase in these two variables can promote or reduce economic growth, and again, what is the effect on economic growth if these two variables (gender inequality and high sex ratio at birth) decrease. In addition, non-linear effects also indicate whether the positive shocks of gender inequality and sex ratio at birth are larger than the negative shocks, or whether the negative shocks of gender inequality and sex ratio at birth are larger than the positive shocks. So for the purpose, this study contributed to the existing literature by examining the non-linear effects of gender inequality and sex ratio at birth on China’s economic growth, using a nonlinear autoregressive distributive lag (NARDL) model, ignoring the traditional ARDL model commonly used in other studies for linear effects. NARDL model is more inclusive and provide robust results taking into account asymmetric trends in time series. Furthermore, the study symmetrically examines the contribution of women to China’s economic growth in terms of labor force participation and education (secondary and higher education).

The remainder of the paper is organized as the next section describes the theoretical and empirical literature review, and Section 3 discusses model construction, data sources, and variable descriptions and methods. Empirical results and their discussion appear in Section 4, namely, “Analysis results and interpretation.” The last section provides concluding remarks and policy implications for the current research.

## Literature review

Gender inequalities and under-empowerment of women hinder their contributions to governance and economic development, as well as improving women’s living standards (Alsaif et al., 2022). In other words, gender equality enables women to gain recognition in health, education, microcredit, and other productive resources (Wei et al., 2021). Gender inequality hinders economic efficiency and growth, reduces quality of life, and ultimately limits productivity (Jackson, 2019; Govindan et al., 2021; Nundy et al., 2021). The level of gender equality is the benchmark for a successful society, and it reflects the level of empowerment and rights of women in that society. Women all over the world are severely marginalized, and both women and men are equally important and have a role to play in social development. According to Quagrainie et al. (2020), women make up half of human resources and they are considered key enablers of sustainable development. According to Heise et al. (2019), gender inequality means discrimination and disparities in the rights, opportunities and responsibilities that all people are entitled to, whether born female or male. Gender disparities in wages, income, skills, wealth, health, and poverty widen differences in developing countries, denying women access to and control over the benefits of economic opportunities and resources. Several reasons were suggested by Ain et al. (2021), Vuong et al. (2021), and Chung and Van der Lippe (2020) argue that gender inequality hinders growth. Gender inequalities and social barriers for all social groups created by economic and social structures hinder sustainable economic growth. Likewise, Syed et al. (2021a) used exploratory factor analysis (EFA), *t*-test, and ANOVA techniques to explore that groups of women in society are more susceptible to psychosocial and organizational stress. The study concludes that females are more socially vulnerable as compared to males. The gender education gap narrows the human capital index, which in turn reduces economic activity and economic growth. Building on foundational work in the late 1980s by Waring and Steinem (1988) and Waring (1999), the broad feminist economics literature increasingly explores the complex interplay between gender inequality and economic growth. The impact of women’s intangible unpaid labor on their rights and autonomy across the country was first noted by Waring. The construction of the Gender Inequality Index (GII) is her work that inspired the United Nations. Gender disadvantage in labor market outcomes, health, and education are key factors affecting long-term economic growth, consistent with Waring’s work on the GII’s three measures. The literature thus explores the impact of gender inequality across multiple dimensions, revealing how the interconnectedness of women’s oppression affects transnational economic development. Several studies have explored the relationship between gender inequality in education and economic growth. And earlier research has shown a positive link between the gender gap in education and economic growth ( Barro and Sala-i-martin 1995; Seguino, 2000; Baliamoune-Lutz and McGillivray, 2009; Elson, 2009; Klasen and Lamanna, 2009), and recent analyses reveal the adverse effects of gender disparities in education on economic growth, using newer data and more careful econometric techniques (Karoui and Feki, 2018; Minasyan et al., 2019; Braunstein et al., 2020; McGee et al., 2020; Perrin, 2021; Santos Silva and Klasen, 2021; Girón and Kazemikhasragh, 2022). Notably, countries with the largest gender gaps lead to greater economic losses. These findings are theoretically consistent, based on the argument that by artificially limiting the talent pool drawn from education, the quality of human capital in society may decline with gender education differences (Klasen and Minasyan, 2017). In the process, countries with constraints on the availability and quality of productive workers may reduce productivity and thus economic growth (Fabozzi et al., 2022; Hickel and Hallegatte, 2022). Furthermore, by promoting female education, the human capital of the next generation can be developed. Higher education stimulates women’s health knowledge, which in turn fosters children’s health (Datu et al., 2021; Diemer et al., 2021). For example, more educated women are positively associated with child health and nutrition, as education increases women’s bargaining power in the household (Alami et al., 2020; Juraqulova and Henry, 2020). In fact, many studies have established that child mortality and adolescent birth rates can be reduced by promoting female education, and economic growth can be boosted by increasing returns on in-kind investments (Keats, 2018). As with the gender education gap, female labor force participation is low and economic growth may stagnate. Elgin and Elveren (2021) use annual cross-country panel data from 1963 to 2018 to uncover the relationship between gender bias employment and economic growth. The results show that gender-biased employment has a significant adverse effect on economic growth in selected panel economies. Furthermore, Klasen and Lamanna (2009) use cross-country and panel regression models to measure the gender gap in employment by examining relative labor force participation rates that significantly reduce economic growth in the Middle East, North Africa, and South Asia. In exploring this relationship, the researchers argue that as countries restrict women’s access to paid employment, average labor costs may increase, reducing their international competitiveness (Lenze and Klasen, 2017; Borrowman and Klasen, 2020; Klasen, 2020).

China’s sex ratio at birth (SRB) has gradually tilted, rising from 108.5/100 women in 1982 to 118.6/100 women in 2005, although it has fallen to 113.5 in 2021 due to the gradual relaxation of family planning policies in recent years. China remains one of the countries in the world with a severe imbalance in the sex ratio at birth (SRB). The disenfranchisement of girls with such abnormally high levels of SRB reflects deep-rooted sexism that adversely affects girls’ development (UNICEF, 2021). Although scholars generally accept the anomalous SRB in China, there is no indisputable conclusion about the contribution of relative causal factors. Female infanticide, the killing of female infants shortly after birth, is one of the leading causes of abnormal sex ratios at birth (SRB) in China. In the 1980s, high female infant mortality due to female infanticide, gender bias in health care and food distribution was the leading cause of high sex ratios at birth (SRB; Chen and Zhang, 2019). In the 1990 census, mortality increased with parity, and high mortality in girls shortly after birth resulted in high SRB (Channon et al., 2021). Another major reason for the high sex ratio at birth is elective abortion in China. Since each family has a fertility quota, pregnancy can only be made within the quota. For example, a family in rural Anhui can have two children. Assessing the likelihood of sex-selective abortion is based on examining approved and unapproved pregnancies separately. Families with child quotas hide their approved pregnancies until the sex of the fetus is known, and if the fetus is female, they unknowingly miscarry (Whittaker, 2022). If the mother conceals her unauthorized pregnancy and stays outside her hometown, the newborn is not registered immediately, but after the mother returns to her hometown (Lai and Choi, 2021). In the 1990s, 70% of late-registered neonates in rural Anhui were male, indicating that sex-selective abortion of female fetuses contributed the most to the extremely high SRB (Chen and Zhang, 2019). From 1986 to 1990, the Chinese government again implemented the tight one-child policy (OCP) nationwide, and the SRB began to rise sharply (National Bureau of Statistics of China, 2020). From 1981 to 2000, the one-child policy was credited with distorting China’s sex ratio, causing approximately 38–48 percent of women (15–20 million) to be infertile. To be more precise, the 4.4% increase in SRB was the result of the implementation of the one-child policy, which contributed 94% to the increase in SRB throughout the 1980s, and the one-child policy increased SRB by about 7, or 57 percent of the increase through the 1990s (Fan et al., 2020). Another fundamental reason for the high gender ratio in China is that son preference has long been reflected in Chinese culture (Nguyen and Le, 2022). There are four main reasons for son preference. First, heavy work requires male labor, especially in rural households. Families without sons are more likely to fall into poverty and various daily difficulties. Second, under the prevailing patriarchal family system, sons support the elderly. Third, a strong motivation for patriarchy is that women wish to improve their status by having sons. Finally, in order to inherit the family business, a son is essential (Marco-Gracia and Beltrán Tapia, 2021).

Overall, women are often neglected by society in terms of labor force participation, health, education, politics, etc., thus widening the gender gap, and female infanticide is one of the main reasons for the abnormal sex ratio at birth in China. As the latest literature above confirms, we could not find any asymmetric studies on the link between gender inequality, sex ratio at birth, and economic growth. Thus, the main contribution of this study to the literature is to empirically explore the asymmetric relationship between gender inequality, sex ratio at birth, and economic growth in China using NARDL techniques covering the period 1980–2020. Moreover, the study empirically examines the contribution of female labor force participation and female education (secondary and higher education) to China’s economic growth.

## Model building, data sources and variable descriptions and methods

### Model specifications

This study adopted the functionalist theory of inequality which believes that society functions so that each individual plays a specific role. Social functioning makes each person play a specific role is the functionalist inequality theory adopted in this study. “Inequality” is the equality necessary for the smooth functioning of society and is the basis for theoretical perspectives and models. Hence, the baseline model of this study is closely related to that of Osabohien et al. (2018) and specified as:


(1) $$Y=f\left(S,M,X,I,E,Z\right)$$

where Y = gross domestic product, S = sex ratio at birth, M = infant mortality rate, I = inequality, E = component of secondary and tertiary education, and Z = female labor force. After incorporating these variables, equation (1) is implicitly specified as:


(2) $$\mathrm{GDP}=f\;\left(\mathrm{SRB},\mathrm{IMR},\mathrm{GIE},\mathrm{FSE},\mathrm{FTE},\mathrm{FLF}\right)$$

The specification of Equation 2 can be explicitly expressed as:


(3) $${\mathrm{GDP}}_{t}=\beta_{0}+\beta_{1}\text{SRBt}+\beta_{2}{\mathrm{IMR}}_{t}+\beta_{3}{\mathrm{GIE}}_{t}+\beta_{4}{\mathrm{FSE}}_{t}+\beta_{5}{\mathrm{FTE}}_{t}+\beta_{6}{\mathrm{FLF}}_{t}+\mu_{i}$$

where GDP is the model dependent variable, representing gross domestic product, used as a proxy for economic growth. GDP, as a proxy for economic growth, is widely used in previous studies by Shabbir et al. (2021), Dabbous and Tarhini (2021), Marozau et al. (2021) and Rahman and Alam (2021). The independent factors are SRB for sex ratio at birth, IMR for infant mortality, GIE for gender inequality, FSE for female secondary education, FTE for female higher education, and FLF for female labor force. β_0_ represents the constant term, β_1_, β_2_…β_6_ are the exogenous variable coefficients, *t* is the time period, and μ_i_ is the random term.

### Variables description, measurement, and data sources

Addressing gender inequality requires a whole-of-government and whole-of-society approach to improve the productivity of life, taking into account the established link between women’s social well-being and economic opportunity (World Health Organization, 2019). The motivation for this study is based on this concept. The study involved seven variables, namely, economic growth peroxides of gross domestic product (GDP), sex ratio at birth, infant mortality rates, inequality, female secondary education, female higher education, and female labor force. Variable inequality data from the United Nations Development Program (UNDP) and remaining variables data from the World Development Indicators (WDI) were obtained for the period 1980–2020. Variable descriptions, measures, and data sources are highlighted in the Supplementary Appendix below.

### Methodology

The appropriate method used in this study to analyze short- and long-term asymmetric relationships between variables is nonlinear autoregressive distributed lag (NARDL). The NARDL model introduced by Shin et al. (2014) works best when the variable integration order is in the level or first order and no variables belong to the second order integration (Gaies et al., 2021; Ghosh and Parab, 2021; Xia et al., 2022). Moreover, bound testing approach employed later in the study as it provides the best results with small sample sizes (Granger and Yoon, 2002; Narayan, 2005).

Most studies only consider linear aspects of the relationship between gender inequality and economic growth, and thus make a significant contribution to the literature (Minasyan et al., 2019; Gavurova et al., 2020); this study analyzes a nonlinear framework for these variables. The nonlinear functional equation based on equation (2) can be written as:


(4) $$\mathrm{GDP}=f\;\left({\mathrm{SRB}}^{+},{\mathrm{SRB}}^{-},{\mathrm{GIE}}^{+},{\mathrm{IEQ}}^{-},\mathrm{FSE},\mathrm{FTE},\mathrm{FLF}\right)$$

The above nonlinear functional equation can be explicitly expressed as:


(5) $$\text{GDPt}=\omega_{0}+\omega_{1}\left({{\mathrm{SRB}}_{t}}^{+}\right)+\omega_{2}\left({{\mathrm{SRB}}_{t}}^{-}\right)+\omega_{3}\left({{\mathrm{GIE}}_{t}}^{+}\right)+\omega_{4}\left({{\mathrm{IEQ}}_{t}}^{-}\right)+\omega_{5}\left(\mathrm{FSE}\right)+\omega_{6}\left(\mathrm{FTE}\right)+\omega_{7}\left(\mathrm{FLF}\right)+\mathrm{\varepsilon i}$$

The model is converted to log-linear form for empirical analysis as follows:


(6) $$\text{lnGDPt}=\omega_{0}+\omega_{1}\ln\left({{\mathrm{SRB}}_{t}}^{+}\right)+\omega_{2}\ln\left({{\mathrm{SRB}}_{t}}^{-}\right)+\omega_{3}\ln\left({{\mathrm{GIE}}_{t}}^{+}\right)+\omega_{4}\ln\left({{\mathrm{IEQ}}_{t}}^{-}\right)+\omega_{5}\ln\left(\mathrm{FSE}\right)+\omega_{6}\ln\left(\mathrm{FTE}\right)+\omega_{7}\ln\left(\mathrm{FLF}\right)+\mathrm{\varepsilon i}$$

where SRB_t_^+^, SRB_t_^−^, GIE_t_^+^, and IEQ_t_^−^ are positive and negative asymmetric variables, showing an asymmetric relationship, and ω_0_, ω_1_, ω_2_, ω_3_, ω_4,_ ω_5,_ ω_6_, and ω_7_ represent long-term parameters.

The short-term effects of variables can be expressed as:


(7) $$\begin{array}{c} \Delta lnGDPt=\kappa_{0}+\sum_{i=1}^{n}\kappa_{1i}\Delta lnGDP_{t-l}+\sum_{i=1}^{n}\kappa_{2i}\Delta lnSRB_{t-i}\\ +\sum_{i=1}^{n}\kappa_{3i}\Delta lnGIE_{t-i}+\sum_{i=1}^{n}\kappa_{4i}\Delta lnFSE_{t-l}\\ +\sum_{i=1}^{n}\kappa_{5i}\Delta lnFTE_{t-i}+\sum_{i=1}^{n}\kappa_{6i}\Delta lnFLP_{t-1}\\ +\rho_{1}lnGDP_{t-1}+\rho_{2}lnSRB_{t-1}+\rho_{3}lnGIE_{t-1}\\ +\rho_{4}lnFSE_{t-1}+\rho_{5}lnFTE_{t-1}+\rho_{6}lnFLP_{t-1}+\varepsilon_{t} \end{array}$$

Equation 7 has been decomposed into short-term and long-term coefficients, κ_1_, κ_2_, κ_3_, κ_4_, κ_5_, and κ_6_ are short-term coefficients, and ρ_1_, ρ_2_, ρ_3_, ρ_4_, ρ_5_, and ρ_6_ are long-term coefficients.

Cointegration regression in a nonlinear framework can be specified as:


(8) $$z_{t}=\alpha^{+}{y_{t}}^{+}+\alpha^{-}{y_{t}}^{-}+\varepsilon_{t}$$

where y_t_ are long-run parameters, which is further decomposed as:


(9) $$y_{t}={y_{t}}^{+}+{y_{t}}^{-}$$

In the equation (9), *y*_t_ is an independent factor, decomposed into a partial sum of positive and negative signs, *y*_t_^+^*y*_t_^−^. The partial decompositions of SRB^t^ and GIE^t^ are highlighted in the following equations.


(10) $$SRB_{t}^{+}=\sum_{i=1}^{k}SRB_{i}^{+}=\sum_{i=1}^{k}max\left(\Delta SRB_{i},0\right)$$

(11) $$SRB_{t}^{-}=\sum_{i=1}^{k}SRB_{i}^{-}=\sum_{i=1}^{k}min\left(\Delta SRB_{i},0\right)$$

(12) $$GIE_{t}^{+}=\sum_{i=1}^{k}IEQ_{i}^{+}=\sum_{i=1}^{k}max\left(\Delta GIE_{i},0\right)$$

(13) $$GIE_{t}^{-}=\sum_{i=1}^{k}IEQ_{i}^{-}=\sum_{i=1}^{k}min\left(\Delta GIE_{i},0\right)$$

The short-term NARDL model based on equation (6) can be specified as:


(14) $$\begin{array}{c} \Delta lnGDP_{t}=\lambda_{0}+\sum_{i=1}^{n}\lambda i\Delta lnGDP_{t-l}+\sum_{i=1}^{n}\lambda i\Delta lnSRB_{t-i}\\ +\sum_{i=1}^{n}\lambda i\Delta lnSRB_{{}_{t-l}}^{-}+\sum_{i=1}^{n}\lambda i\Delta lnGIE_{t-i}^{}\\ +\sum_{i=1}^{n}\lambda i\Delta lnGIE_{t-l}^{-}+\beta_{1}lnGDP_{t-l}+\beta_{2}lnSRB_{t-l}\\ +\beta_{3}lnSRB_{t-1}^{-}+\beta_{4}lnGIE_{t-l}+\beta_{5}lnGIE_{t-l}^{-}+\mu_{i} \end{array}$$

## Analysis results and interpretation

Table 1 highlights the descriptive statistics of the proposed model variables, indicating that $1,191.2 billion is the average GDP of China and show substantial variation as represented by its SD value. The mean sex ratio at birth is 1.52, reflecting 1.52 boys born for every one girl. The average infant mortality rate is 21, indicating an average of 21 deaths per 1,000 live births. The average gender inequality is 0.52, reflecting that 52% of men prioritized basic human rights over women. Likewise, female secondary education and female tertiary education averaged 67.36 and 35.31, respectively, replicating female enrolment rates at these two stages of education. Finally, 57.57 is the average female labor force participation rate, indicating that 57% of women are likely to work and participate in the labor force. Furthermore, the Jaque-Bera test probability for all variables is higher than 10%, which show that all variable data are normally distributed. Variable positive statistics in skewness indicate that all variables are positively skewed. Kurtosis shows that GDP is lanky and peaking due to high statistics.

**Table 1:** Descriptive statistics.

		lnGDP	lnSRB	lnIMR	lnGIE	lnFSE	lnFTE	lnFLF
Mean		11,912	1.52	21	0.51	67.36	35.31	57.57
Median		11,781	1.45	23	0.55	68.32	33.39	58.41
Maximum		21,287	1.92	38	0.75	91.54	69.52	91.43
Minimum		7,213	1.07	5	0.32	33.81	4.58	52.67
SD		10,234	0.62	21	0.35	19.37	55.36	43.31
Kurtosis		1.9	1.41	1.18	1.27	1.49	1.74	1.63
Skewness		3.2	0.39	0.71	0.29	0.71	0.83	0.73
Jarqua-Bera		2.1	1.37	1.48	1.38	1.63	1.74	1.83
Probability		0.60	0.68	0.79	0.82	0.92	0.56	0.63

The nonlinear autoregressive distributed lag model (NARDL) proposed by Shin et al. (2014) used in this study has various advantages over other cointegration models. Using this model produces robust results when the variables integration order is mixed and the data are for small samples size. Stationarity checks are not mandatory for applying NARDL models, as suggested by previous studies (Abbasi et al., 2022; Amin et al., 2022). However, as highlighted by some studies, this model is not suitable for second-order integrals because the results of the bound F statistic become invalid in the case of I (2; Alqahtani et al., 2020; Syed, 2021a,b; Syed et al., 2021b, 2022; Bertsatos et al., 2022; Xia et al., 2022). Hence, this study used three different unit root tests, the DF-GLS test proposed by Elliot et al. (1996), Augmented Dickey Fuller (ADF) Dickey and Fuller (1981), and Phillips and Perron (PP) Phillips and Perron (1988) to test variable integrals. Criticized for low power of ADF and PP tests when variables are stationary but roots are close to non-stationary boundaries (Dogan and Seker, 2016). Elliot et al. (1996) considered the DF-GLS test to be more powerful than the ADF and Phillips-Perron tests in the presence of unknown mean or trend.

The results of the ADF, PP, and DF-GLS tests, shown in Table 2, indicating that all variables have unit roots at levels but integrate at the first difference of I(1), and none of the variables integrate at I(2).

**Table 2:** ADF, PP, and DF-GLS unit root test.

	ADF test		PP test		DF-GLS test	
	Level I(0)	First difference	Level I(0)	First difference	Level I(0)	First difference
lnGDP	−0.342	−1.485^*^	−0.425	−1.284^*^	−0.435	−1.209^*^
lnSRB	−0.273	−1.334^*^	−0.325	−1.684^*^	−1.384	−2.918^*^
lnGIE	−0.362	−1.326^*^	−1.436	−1.687^*^	−1.249	−3.214^*^
lnFSE	−0.232	−1.263^*^	−0.453	−1.436^*^	−1.343	−1.491^*^
lnFTE	−0.324	−1.426^*^	−0.534	−1.328^*^	−0.435	−1.286^*^
lnFLF	0.426	1.358^*^	0.624	1.326^*^	−1.536	−2.625^*^
lnIMR	0.602	1.392^*^	0.343	1.975^*^	−2.928	−3.218^*^

* denotes null hypothesis rejection at significance level of 1%

** denotes null hypothesis rejection at significance level of 5%.

*** denotes null hypothesis rejection at significance level of 10%.

Following the studies of Ullah et al. (2021) and Qi et al. (2022), the BDS test proposed by Brook et al. (1996) can be used to explore non-linear dependencies in the proposed variable data. The BDS test is able to highlight model error specifications while being compared to other nonlinear tests and capture nonlinear properties that other tests ignore. The data are independent and identically distributed (i.i.d) is the null hypothesis of the BDS test. If the null hypothesis is rejected, a linear model cannot be applied (as is the case in this study), thereby confirming nonlinear dependencies in the series and validating the applicability of the nonlinear ARDL (NARDL) method. The BDS test results are shown in Table 3, which clearly show that the significance of the BDS test probability value is at the 1% level, confirming that the data are not linear.

**Table 3:** BDS test for detecting nonlinear dependencies.

BDS statistics	Embedding dimensions = m			*m* = 2	*m* = 3	*m* = 4	*m* = 5	*m* = 6
lnGDP	0.3304^*^	0.3418^*^	0.3975^*^	0.4437^*^	0.5464^*^
lnSRB	0.3684^*^	0.4891^*^	0.5365^*^	0.5467^*^	0.6849^*^
lnGIE	0.4917^*^	0.4164^**^	0.5478^*^	0.6433^*^	0.6854^**^
lnFSE	0.5458^*^	0.5964^*^	0.4686^**^	0.3854^*^	0.5461^*^
lnFTE	0.3681^***^	0.4358^**^	0.5342^***^	0.3841^**^	0.4389^**^
lnFLF	0.3841^*^	0.4563^*^	0.5643^*^	0.6193^**^	0.4376^*^
lnIMR	0.4952^**^	0.5647^*^	0.5754^**^	0.7204^**^	0.5487^*^

* denotes null hypothesis rejection at significance levels of 1%.

** denotes null hypothesis rejection at significance level of 5%.

*** denotes null hypothesis rejection at significance level of 10%.

Previous research has shown that optimal lag selection has a large impact on long-term outcomes (Guan et al., 2020; Wu and Xie, 2020). Model estimation can lead to erroneous conclusions with less lag selection; however, higher lag selection can lead to overestimation of results. Thus, two lag lengths were selected based on the *SIC* criterion of the optimal lag length. Going a step further, the ARDL bound test method was used first; as shown in Table 4, in the linear ARDL specification, the lower and upper bounds of the proposed model are 2.64 and 3.87, respectively, at the 5% significance level. The F statistic of Pesaran et al. (2001) is 2.01, which is lower than the corresponding upper and lower bounds, thus clearly verifying that there is no cointegration between GDP and explanatory variables. The NARDL bound testing approach is then used to examine long term asymmetric relationships between the variables of interest in the proposed model. At the 5% significance level, the lower and upper bounds of the nonlinear ARDL specification are 2.31 and 3.54, respectively. The F statistic of Pesaran et al. (2001) is 5.898, which is above the upper and lower bounds, thus confirming long-term cointegration. The NARDL bound test model results predicted the likelihood of asymmetric long-term relationships among the proposed variables.

**Table 4:** ARDL and NARDL bound testing approaches for cointegration.

	F-stat	Lower-upper Bound (1%)	Lower-upper Bound(5%)	Lower-upper Bound(10%)	K	Result
*InGDP/(InSRB, InGIE, InFSE InFTE, InFLF, InIMR)*	2.01	3.43–4.51	2.64–3.87	2.45–3.47	6	No co-integration
*InGDP/(InSRB^+^, InSRB^−^, InGIE InGIE^−^, InFTE, InFLF, InIMR)*	5.898^***^	3.10–4.28	2.31–3.54	2.37–3.42	6	Co-integration

* is the significant level at 10%.

** is the significant levels at 5%.

*** is the significant level at 1%.

The estimated NARDL long-term coefficient results are shown in Table 5. The main purpose of this study is to examine the asymmetric relationship between gender inequality, sex ratio at birth, and economic growth, as well as to explore the association between other important explanatory variables and economic growth. The long-term effects of the estimated coefficients are both positive and negative for both decrease and increase in economic growth. The estimated coefficients for the sex ratio at birth (SRB) are +0.679 and-0.668, respectively, suggesting that for every 1% increase in the sex ratio at birth, economic growth is expected to decline significantly by 0.668%, while a 1% decrease in the sex ratio drives economic growth significantly by 0.679%. This finding is very consistent with the work of Schacht et al. (2019), Chao et al. (2020), and Grech (2018). Likewise, the estimated coefficients for gender inequality are +0.572 and-0.598, respectively, indicating that a 1% increase in gender inequality is expected to significantly reduce economic growth by 0.598%, while a 1% reduction in gender inequality can significantly boost economic growth by 0.572%. The finding of the negative and significant impact of gender inequality on economic growth is in good agreement with those of Kim et al. (2018), Altuzarra et al. (2021), Santos Silva and Klasen (2021), McGee et al. (2020), Tisdell (2021), Gavurova et al. (2020) and Karoui and Feki (2018). The Wald statistic confirms the long-run asymmetry by rejecting the null hypothesis that gender inequality and sex ratio at birth have symmetric effects on economic growth. The coefficients of female secondary education, female tertiary education, and female labor force participation are 0.354, 0.465, and 0.362 respectively, indicating that female secondary education, and female labor force participation rate can significantly boost economic growth by more than 35%, and female higher education boosts economic growth by over 45%. The result clearly shows that, in the long run, positive sex ratio at birth shocks has a lower impact on economic growth than negative shocks. And the positive gender inequality shocks have a higher impact on economic growth in the long run than negative shocks.

**Table 5:** NARDL long-term variable elasticities results (Dependent variable: GDP).

Variables	Coefficient	Standard error	*t*-statistics	Probability
In(SRB)^+^	−0.668^***^	0.116	−4.024	0.003
In(SRB)^−^	0.679^***^	0.134	3.300	0.012
In(GIE)^+^	−0.598^***^	0.422	−5.276	0.000
In(GIE)^−^	0.572^**^	0.477	4.035	0.002
InFSE	0.354^***^	0.062	6.015	0.000
InFTE	0.465^***^	1.062	6.274	0.000
InFLF	0.362^**^	1.662	2.215	0.029
InIMR	−0.284^***^	0.436	−4.465	0.001
Constant	−6.834^***^	1.623	−7.345	0.000
R^2^	0.99			
Adj R^2^	0.81			
F-statistic	623.74			
Wald statistic 1.092 (0.141)				

* is the significant level at 10%.

** is the significant levels at 5%.

*** is the significant level at 1%.

Exploring the short-run elasticity between GDP and explanatory variables, again using the *SIC* criterion of optimal lag length to choose lag length 1. The NARDL short run elasticities are presented in Table 6. Based on long-term elasticity, short-term estimates also show that the elasticity coefficients for gender inequality and sex ratio at birth are decomposed into positive and negative ones, respectively. In the model specification, the coefficients are −0.659 and + 0.583, respectively, which indicates that every 1% increase in the sex ratio at birth is expected to significantly reduce economic growth by 0.659%, while every 1% decrease in sex ratio at birth is expected to significantly boost economic growth by 0.583%. Likewise, the coefficients −0.522 and 0.559 indicate that a 1% increase in gender inequality significantly reduces economic growth by 0.522%, while a 1% reduction in gender inequality significantly increases economic growth by 0.559%. Wald test rejects the null hypothesis of symmetric effects by confirming the asymmetry. Looking at the results of other explanatory variables, female secondary education, female higher education, and female labor force participation rate have a driving effect on short-term economic growth. The progressive effect of female secondary education and female labor force participation on economic growth is not significant, but the effect of female higher education is significant. Infant mortality has a significant adverse effect on economic growth. From this analysis, few important points are noted. First, comparing the short- and long-term corresponding elasticities of sex ratio at birth to gender inequality shows that the long term elasticities are statistically higher in magnitude. Second, the positive and negative components of the long- and short-run elasticities of sex ratio at birth and gender inequality are both inverse and statistically significant for economic growth. Third, both the long- and short-term elasticities of sex ratio at birth are higher than the corresponding elasticities of the gender inequality.

**Table 6:** NARDL short-term variable elasticities results (Dependent variable: GDP).

Variables	Coefficient	Standard error	t-statistics	Probabilityty
∆In(SRB)^+^	−0.659^**^	0.127	−2.024	0.043
∆In(SRB)^−^	0.583^**^	0.145	2.010	0.040
∆In(IEQ)^+^	−0.522^***^	0.533	−5.387	0.000
∆In(IEQ)^−^	0.559^***^	0.588	4.145	0.002
∆InFSE	0.463	0.283	1.032	0.172
∆InFTE	0.115^*^	0.284	1.974	0.050
∆InFLF	0.473	1.773	1.326	0.129
∆InIMR	−0.315^***^	0.117	−5.576	0.001
ECM(−1)	−0.545^***^	1.734	4.456	0.000
*R* ^2^	0.92			
Adj *R*^2^	0.95			
D-W statistic	4.449			
Wald statistic	1.214 (0.263)			

* is the significant level at 10%.

** is the significant levels at 5%.

*** is the significant level at 1%.

Thus, considering these facts, we conclude that the long-term effects of sex ratio and gender inequality at birth in China are stronger than the short-term, as the effects become stronger over time. The error correction mechanism (ECM) coefficient is −0.545, indicating that sex ratio at birth and gender inequality adjust to balance at a rate of 54% in the presence of other variables. *R*-squared values of 0.99 and 0.92 are lower than the Durbin-Watson statistic of 4.449, confirming that there is no spurious regression problem in the model. The diagnostic test results in Table 7 confirm the absence of serial correlation and heteroskedasticity issues, and the model passes other tests such as the Jarque-Bera normality test, Breuch-Pagan-Godfrey test, ARCH, and Ramey Reset.

**Table 7:** Diagnostic tests for the NARDL model.

Diagnostic Tests	F-statistics	Probability
Normality (Jerque-Bera) test		8.352	0.425
Serial correlation	0.8613	0.655
Breuch-Pagan-Godfrey test		1.2515	0.527
ARCH	0.3694	0.962
Ramey Reset	1.3995	0.460

Model stability was checked using the CUSUM and CSUSMQ tests, and the results in Supplementary Appendix B show that the model is stable because the estimated line lies within the boundaries of the critical line at the 5% significance level.

Dynamic multiplier plots were used to examine asymmetries due to positive and negative shocks to sex ratio at birth and gender inequality. As shown in Supplementary Appendix C, the curves display evidence of asymmetric adjustment for positive and negative shocks in the long-run equilibrium of sex ratio at birth and gender inequality. The graph also shows that, in the long run, positive sex ratio at birth shocks has a lower impact on economic growth than negative shocks. The graph also shows that positive gender inequality shocks have a higher impact on economic growth in the long run than negative shocks.

## Concluding remarks

China has some of the worst gender inequality in the areas of economic, education, health, and politics. Among the 153 countries with the smallest to worst overall gender gap, China ranks 106th. China ranks 91st out of 153 countries for the gender gap in economic participation and opportunity, lower than emerging economies such as Brazil and Russia (World Economic Forum, 2020). At a time when growth is already slowing, the widening gender gap in China’s labor market—if it persists—could become an even bigger burden on the economy. China’s rise as a global economic power over the last few decades has put women at a disadvantage and worsened gender inequality in its workforce. China’s rise as a global economic powerhouse over the past few decades has disadvantaged women and exacerbated gender inequality in the workforce. Female labor force participation rates have fallen to low levels by international standards, gender pay gaps, and gender discrimination are pervasive in the labor market, and there is evidence of growing prejudiced perceptions of women’s rights at work and workplace leadership. Women’s economic empowerment, increased productivity, income equality, and economic diversification are central to achieving women’s rights and gender equality, among other positive development outcomes. Higher education for women and girls contributes to more inclusive economic growth and the economic empowerment of women. Education, upskilling, and retraining across the lifespan, especially to keep up with the rapid technological and digital transformation affecting employment, is essential for the health and well-being of women and girls, as well as their income-generating opportunities and participation in the formal education workforce. China remains one of the countries in the world with a severe imbalance in the sex ratio at birth (SRB). The disenfranchisement of girls with such abnormally high levels of SRB reflects deep-rooted sexism that adversely affects girls’ development. Female infanticide, the killing of female infants shortly after birth, is one of the leading causes of abnormal sex ratios at birth (SRB) in China. High female infant mortality due to female infanticide, gender bias in health care, and food distribution was the leading cause of high sex ratios at birth (SRB). Another major reason for the high sex ratio at birth is elective abortion in China. Since each family has a fertility quota, pregnancy can only be made within the quota.

The present study empirically predicts an asymmetric relationship between gender inequality, sex ratio at birth, and economic growth, using NARDL model over the period 1980–2020. The NARDL results show that increases in gender inequality and sex ratio at birth significantly reduce economic growth in both the short and long term, while reductions in gender inequality and sex ratio at birth significantly boost economic growth in both the short and long term. First, comparing the short- and long-term corresponding elasticities of sex ratio at birth to gender inequality shows that the long term elasticities are statistically higher in magnitude. Second, the positive and negative components of the long- and short-run elasticities of sex ratio at birth and gender inequality are both inverse and statistically significant for economic growth. Third, both the long- and short-term elasticities of sex ratio at birth are higher than the corresponding elasticities of the gender inequality. Moreover, the study explored the significant contribution of female labor force participation and female education (secondary and higher education) to economic growth. However, infant mortality significantly reduced economic growth.

Women are an integral part of society, making up half of human capital and key to sustainable development and quality of life. So they should be members of the community center. People in society should treat daughters and sons equally. Men and women are equally important and play a role in social development. This research helps to provide eye-opening insights into the links between gender inequality, sex ratio at birth and economic growth in China. Strategically, the study recommends equal opportunities for women in employment, education, health, economics and politics to reduce gender disparities and thereby promote sustainable economic growth in China. This study prioritizes women’s access to education, educating women like educating families, they are more likely to participate equally in the workforce, lead healthier, more productive lives, and become decision makers in families and communities, thereby promoting economic growth. Moreover, policymakers should introduce new population policy to stabilize the sex ratio at birth, thereby promoting China’s long-term economic growth.

Regarding study limitations, this study did not examine the link between gender inequality in women’s political participation and economic growth, so future research needs to explore the link between gender inequality in women’s political participation and economic growth. Moreover, this analysis is for a single country, we recommend panel data analysis for future studies to obtain broader conclusions, using the NARDL method for countries with a higher sample.

## Data availability statement

Publicly available datasets were analyzed in this study. This data can be found here: World Bank Development indicators, https://datacatalog.worldbank.org/dataset/world. UNDP Gender Inequality Index (GII), https://hdr.undp.org/data-center/thematic-composite-indices/gender-inequality-index#/indicies/GII.

## Author contributions

AA and XW contributed to the conceptualization of the study, analysis, design, and conclusions, reviewed the manuscript, and approved the final submission. WH, TZ, and JC conceptualized and revised the study, software data curation, editing, and literature search. All authors contributed to the article and approved the submitted version.

## Conflict of interest

WH was employed by company China Everbright Group.

The remaining authors declare that the research was conducted in the absence of any commercial or financial relationships that could be construed as a potential conflict of interest.

## Publisher’s note

All claims expressed in this article are solely those of the authors and do not necessarily represent those of their affiliated organizations, or those of the publisher, the editors and the reviewers. Any product that may be evaluated in this article, or claim that may be made by its manufacturer, is not guaranteed or endorsed by the publisher.

## Supplementary material

The Supplementary material for this article can be found online at: https://www.frontiersin.org/articles/10.3389/fpsyg.2022.1003467/full#supplementary-material
